This article has been retracted.

# The Effect on the Fracture Healing following Femoral Neck Shortening after Osteoporotic Femoral Neck Fracture Treated with Internal Fixation: Finite Element Analysis

**DOI:** 10.1155/2021/3490881

**Published:** 2021-08-04

**Authors:** Xiao Yu, Peng-ze Rong, Qing-jiang Pang, Xian-jun Chen, Lin Shi, Cheng-hao Wang

**Affiliations:** ^1^Department of Orthopedics, HwaMei Hospital, University of Chinese Academy of Sciences; Ningbo Institute of Life and Health Industry, University of Chinese Academy of Sciences, Ningbo 315000, China; ^2^Ningbo University School of Medicine, Ningbo 315211, China

## Abstract

**Objective:**

To evaluate the stress status of fracture site caused by femoral neck shortening and to analyze the stress of fracture site and the implants from the finite element point of view.

**Methods:**

CT scan data of hip of a normal adult female were collected. Three-dimensional reconstruction MICs and related module function simulation was used to establish the postoperative shortening model of femoral neck fracture with Pauwels angle > 50°, which was treated with cannulated screws. The models were divided into four groups: normal femoral neck, shortening in 2.5 mm, shortening in 7.5 mm, and shortening in 12.5 mm. The finite element analysis software msc.nastran2012 was used, and the data of maximum stress and stress nephogram of fracture site and implants were carried out.

**Results:**

From normal femoral neck to shortening in 12.5 mm of the femoral neck, the maximum tensile stress increased gradually in the fracture site above the cannulated screws while compressive stress decreased gradually in the fracture site below the cannulated screws, and the maximum stress of the cannulated screws increased gradually with obvious stress concentration at the screw holes in the fracture site, and the peak value of stress concentration was about 179 MPa.

**Conclusion:**

The biomechanical environment of the fracture site changed by femoral neck shortening. With the increasing of femoral neck shortening, the stress of the fracture site and implants would be uneven; then, the stability of fracture site would become worse, and the possibility of implant sliding or even breakage would be increased.

## 1. Introduction

Femoral neck fracture is a senile disease. However, the fracture in 60-65 years old is usually treated by internal fixation with cannulated screws, which was considered as an important method to preserve the hip joint [1, 2]. However, due to the situation such as osteoporosis, it is not uncommon to see the femoral neck shortening after cannulated screw placement [3]. The shortening of the femoral neck will inevitably cause the shortening of the lower limb, which will change the patient's gait. For a long time, it will affect the abduction function of hip joint and pelvic stability, thus affecting the quality of life [4, 5]. Some scholars reported their researches about the stability of the femoral neck fracture fixation by finite element analysis and the comparison with the dynamic hip screw and cannulated screws by biomechanical evaluation [6–8]; however, there was few biomechanical experiment to verify the biomechanical effect of neck shortening on fracture healing after internal fixation with cannulated screws. In fact, it is necessary to understand the biomechanical effect, which helps the surgeons to judge what kind of degree of shortening needs early intervention. It has been confirmed that femoral neck shortening after internal fixation with cannulated screws will significantly reduce the Harris score of hip joint due to the abnormal gait of claudication of the injured limb and limitation of the abduction of the injured hip [9–12]. Therefore, this study aims to establish a three-dimensional model of femoral neck fracture with cannulated screw fixation and analyze the stress distribution and changes on the fracture site and implants by finite element method, so as to explore the biomechanical effect of femoral neck shortening on fracture healing after internal fixation of femoral neck fracture.

## 2. Material and Method

### 2.1. The Establishment of Normal Hip Joint Model and Femoral Neck Fracture Model with Neck Shortening

A 60-year-old female volunteer, 160 cm in height and 55 kg in weight, was randomly selected in the hospital. The abnormal conditions such as necrosis of the femoral head, acetabular defect and dysplasia, and hip joint disease were excluded by X-ray examination. The patient was diagnosed as osteoporosis by dual energy X-ray absorptiometry (DXA). The study was approved by the ethics committee in the hospital, and the volunteers signed the informed consent before the examination.

The volunteer was supine on the CT bed, and the lower extremities were in the neutral position. The hip joint was scanned from the upper edge of the acetabulum to the middle part of the femoral shaft. After scanning, the CT image data of 512 × 512 matrix, 260 layers in total, was obtained, and the scanned data was stored directly in Dicom format. The Dicom files were loaded into software of Mimics 16.0. The original images were set in the directions of front, back, left, and right and accurately matched the orientation of the reconstructed 3D model with the human body coordinate axis. The osseous tissue was extracted by threshold method with the range of 122-1613 Hu. The extracted tissue was stored in a mask, and the pixels in the mask were modified by mask editing, region growing, and cavity filling. Then, the STL file was loaded into the software of Geomagic studio 2014, which could build a watertight nonuniform rational spline curve and could be optimized for surface fitting and fairing. It could be curved through the process of accurate surface and finally formed a three-dimensional solid model of the hip joint, which was conducive to the subsequent finite element model establishment and analysis (Figure 1).

## 3. The Model Assembly

In order to facilitate the establishment of hip joint finite element model and data processing, the implant size was referred to the operation of internal fixation of femoral neck fracture. Three cannulated screws (Synthes, Swiss) were commonly used with the screw diameter 4.8 mm, thread diameter 7.3 mm, and hollow diameter 2.6 mm. However, the screw length was depended on the actual length of the femoral neck. The cannulated screws were arranged in an inverted triangle, and the thread shape of the screw was ignored in the process of screw modeling. The contact setting was used in the calculation process to achieve a good contact between the thread of the cannulated screws and the femoral neck. It was assumed that the femoral neck was complete fracture and had been anatomical reduction. The Pauwels angle was more than 50°, and the friction coefficient between the two fracture surfaces was 0.15. The relationship between the femoral neck and the thread of the cannulated screws was set as binding without displacement; however, the relationship between the screw paths and the unthreaded part of the screws was set as contact, and the friction coefficient was 0.2. The shortening model of femoral neck after internal fixation could be completely obtained. According to the shortening length, the models could be divided into four groups: no femoral neck shortening model (0 mm), mild shortening model (2.5 mm), moderate shortening model (7.5 mm), and severe shortening model (12.5 mm) (Figure 2).

## 4. Generating the Finite Element Model and Assigning Material to the Model

The IGES files of four groups of the models were imported into HyperMesh 13.0 software for mesh generation, the BDF format files were then exported, and the finite element postprocessing calculation and analysis were carried out in msc.nastran2012 software.

The modulus of elasticity and Poisson's ratio were selected as the parameters of material assignment. The femur is made up of cancellous bone, cortical bone, and hollow medullary cavity, and it has the characteristics of heterogeneity and belongs to anisotropic nonlinear body. Therefore, we referred to the published research data [13–15], titanium alloy (Ti6Al4VELI) material was used for the cannulated screws, and the material parameters of the model were listed in the table below (Table 1).

## 5. Constraint Condition and Mechanical Loading

The boundary constraint conditions for four groups of the models were hypothesized: (1) it was assumed that a distal femoral fixation constraint and the degrees of freedom in six directions for all nodes on the distal of femur are limited. (2) It was assumed that the structure of femur is a continuous, uniform, and isotropic linear elastic material [15]. In this study, the commonly used simplified model was adopted, the peak force of the single hip was tested when the 55 kg volunteer was walking normally, and the joint was loaded at the peak time [15]. The reaction resultant of the hip joint force was about 2072 N, and abductor muscle resultant force was about 8737 N. The resultant joint forces are distributed in a cosine fashion on the surface of the femoral head [15]. The model of assigned material was imported into the finite element analysis software Msc.Nastran2012 and loaded the constraints, and then, the calculation and analysis could be carried out (Figure 3).

## 6. Results

### 6.1. Finite Element Simulation of Cannulated Screws with Different Degree of Femoral Neck Shortening

From normal femoral neck without shortening to shortening in 2.5 mm, 7.5 mm, and 12.5 mm of the femoral neck, the maximum tensile stress of cannulated screws in the fracture site above femoral neck were 115.2 MPa, 117.3 MPa, 120.0 MPa, and 136.6 MPa, respectively; however, the maximum compressive stress of cannulated screws in the fracture site below the femoral neck were 12.4 MPa, 12.3 MPa, 10.9 MPa, and 9.4 MPa, respectively. It demonstrated that with the increase of the shortening, the maximum stress of the cannulated screws gradually increased, and there was an obvious stress concentration at the fracture site on the cannulated screws. The peak stress of three cannulated screws were 237.4 MPa, 237.6 MPa, 256.4 MPa, and 276.5 MPa, respectively, which meant that it might the place with high incidence of stress fatigue of the implants in clinical application (Figure 4).

## 7. Finite Element Simulation of Fracture Site with Different Degree of Femoral Neck Shortening

From normal femoral neck without shortening to shortening in 2.5 mm,7.5 mm, and 12.5 mm of the femoral neck, the maximum compressive stress of the medial bone of the femoral neck were 19.9 MPa, 18.8 MPa, 4.0 MPa, and 2.1 MPa, respectively, while the maximum compressive stress of the lateral bone of the femoral neck were 31.7 MPa, 32.5 MPa, 34.2 MPa, and 36.8 MPa, respectively. The maximum stress at the fracture site of femoral neck was 152.2 MPa, 159.3 MPa, 161.4 MPa, and 179.2 MPa, respectively. It demonstrated that with the increase of the shortening, the tensile stress of two screws above the femoral neck increased, while the compressive stress under the femoral neck decreased. It also demonstrated that the stress on the fracture site increased gradually (Figure 5). When the fracture was not healed, the increased stress might augment the possibility of implant sliding and breakage, especially in the osteoporotic patients, which the implant might bear the additional stress and subsequently affect the stability of the fracture site and increase the difficulty of fracture healing [16, 17].

## 8. Discussion

In recent years, the treatment of femoral neck fracture with cannulated screw has become a better method with satisfied clinical effect [18, 19]. However, neck shortening often occurs after internal fixation with cannulated screw, especially in the osteoporotic population [19]. Some clinical studies have shown that the osteoporotic femoral neck fracture, especially for the cases of neck shortening can significantly reduce the Harris score of hip joint. For example, Bartels et al. [20] pointed out that patients aged 55-70 years with a displaced femoral neck fracture might have lower bone density, higher comorbidity, and subsequently the worse function of the hip. Another example was that Chen et al. [21] compared DHS-BLADE and cannulated compression screws in the treatment of femoral neck fractures and found that the DHS-BLADE had advantages over cannulated compression screws for preventing femoral neck shortening, screw migration, and cut-out, which might keep the function of the hip in a high place. However, there is no strict biomechanical experiment to study the biomechanical effect of femoral neck shortening on the healing of femoral neck. We classify the different degrees of femoral neck shortening and divided it into four types by modeling in finite element method: normal group (without shortening), shortening mild group (shortening 2.5 mm), moderate group (shortening 7.5 mm), and severe group (shortening 12.5 mm). The stress of cannulated screw and fracture site were simulated by mechanical loading [22].

In this study, the maximum stress of three cannulated screws in four groups was increased with the increase of neck shortening. In addition, from the stress nephogram of the femoral neck, the stress concentration was obvious at the fracture site on the cannulated screws, which meant that it might the place with high incidence of stress fatigue of the implants in clinical application. It is normal to produce stress concentration because of the loading to the femoral neck in the condition of slow walking, which will lead to the extrusion between the cannulated screws and the femoral neck, so it is easy to produce stress concentration near the screw holes. At present, the yield strength of titanium alloy for implant material is about 817 MPa [22]; therefore, from this point of view, the internal fixation structure of three cannulated screws after neck shortening is still within the range of yield strength. However, the stress of implants in this experiment was measured under the condition of slow walking, which was different from the maximum stress produced by the actual movement after the operation of femoral neck fracture, so there was still a risk of breakage of cannulated screws in stress concentration. Some scholars have established the finite element model of the femoral neck shortening after internal fixation of the femoral neck fracture and found that the residual screw holes of the cannulated screws will reduce the quality of the bone structure [23]. Meanwhile, due to the loss of the support protection of the cannulated screws, the risk of fracture will be greatly increased after the removal of the cannulated screws [24].

The results also showed with the increase of the shortening, the tensile stress of two screws above the femoral neck increased, while the compressive stress under the femoral neck decreased. It also demonstrated that the stress on the fracture site increased gradually, which increased the possibility of internal fixation sliding, thus affecting the stability of the fracture site and increasing the difficulty of fracture healing. Therefore, from the biomechanical point of view, excessive stress on the fracture site might aggravate the shortening of the femoral neck, which is not conducive to the healing of the fracture, especially in the osteoporosis population. Furthermore, the shortening of femoral neck after cannulated screw fixation would affect the activity and function of hip joint and the Harris score of hip joint would decrease [25].

In summary, the healing of femoral neck fracture requires a stable environment constructed by compression between the fracture site [18, 26]; however, the shortening of the femoral neck caused by the compression between the fracture sites should not be ignored as we stated above. The increased shortening of the femoral neck will also lead to instability of fracture, increase the risk of implants breakage, and even cause the hip joint dysfunction [27]. It is suggested that we should pay attention to the effect of “excessive” compression which might cause the femoral neck shortening.

## Figures and Tables

**Figure 1:** Geometric models and the cannulated screws retreat in different femoral neck shortening after cannulated screws fixation. (a) No shortening, (b) shortening in 2.5 mm, (c) shortening in 7.5 mm, and (d) shortening in 12.5 mm; 1: geometric models and 2: cannulated screws retreat.

**Figure 2:** The models of shortening after internal fixation of femoral neck in four groups. (a) No shortening, (b) shortening in 2.5 mm, (c) shortening in 7.5 mm, and (d) shortening in 12.5 mm.

**Figure 3:** Boundary constraints of femoral neck shortening model.

**Figure 4:** Von Mises stress diagram of cannulated screws with different degrees of femoral neck shortening. (a) No shortening, (b) shortening in 2.5 mm, (c) shortening in 7.5 mm, and (d) shortening in 12.5 mm.

**Figure 5:** Von Mises stress maps and equivalent strain maps of femoral neck fractures with different shortening of femoral. (a) No shortening, (b) shortening in 2.5 mm, (c) shortening in 7.5 mm, and (d) shortening in 12.5 mm; 1: von Mises stress maps and 2: equivalent strain maps.

**Table 1:** The material parameters of femoral neck shortening model after cannulated screw fixation.

Structural region	Modulus of elasticity (MPa)	Poisson's ratio
Cortical bone of femur	16 800	0.30
Cancellous bone of femur	620	0.29
Acetabular cartilage	10	0.40
Cannulated screw (Ti6Al4VELI)	110 000	0.33

## Data Availability

The data used to support the findings of this study are available from the corresponding author upon request.
